RETRACTED

# E2F1 Affects the Therapeutic Response to Neoadjuvant Therapy in Breast Cancer

**DOI:** 10.1155/2022/8168517

**Published:** 2022-09-17

**Authors:** Xinxing Ye, Jie Zhou, Dandan Tong, Dandan Wang, Hui Wang, Jixue Guo, Xinmei Kang

**Affiliations:** ^1^Department of Medical Oncology, The Second Hospital of Harbin, Harbin, Heilongjiang Province, China; ^2^Department of Medical Oncology, Xiang'an Hospital of Xiamen University, School of Medicine, Xiamen University, Xiamen, Fujian Province, China; ^3^School of Medicine, Huaqiao University, Quanzhou, Fujian Province, China; ^4^Department of Medical Oncology, Heze Peony People's Hospital, Heze, Shandong Province, China; ^5^Department of Medical Oncology, Shandong Cancer Hospital Affiliated to Shandong University, Shandong Province, China; ^6^Department of Medical Oncology, Heilongjiang Provincial Hospital, Harbin, Heilongjiang Province, China

## Abstract

This study is aimed at screening genes for predicting the sensitivity response and favorable outcome of neoadjuvant therapy in breast cancer. We downloaded neoadjuvant therapy genetic data of breast cancer and separated it into the pathological complete response (pCR) group and the non-pCR group. Differential expression analysis was performed to select the differentially expressed genes (DEGs). After that, we investigated the enriched biological processes and pathways of DEGs. Then, core up/down protein-protein interaction (PPI) network was, respectively, constructed to identify the hub genes. A transcription factor-target gene regulation network was built to screen core transcription factors (TFs). We found one upregulated DEG (KLHDC7B) and four downregulated DEGs (TFF1, LOC440335, SLC39A6, and MLPH) overlapped in three datasets. All DEGs were mainly enriched in pathways related to DNA biosynthesis, cell cycle, immune response, metabolism, and angiogenesis. The hub genes were KRT18, IL7R, HIST1H1A, and E2F1. The core TFs were HOXA9, SPDEF, FOXA1, E2F1, and PGR. RT-qPCR suggested that E2F1 was overexpressed in MCF-7, but HOXA9 was low-expressed. Western blot suggested that the MAPK signal pathway was inhibited in MCF-7/ADR. That is to say, some genes and core TFs can predict the sensitivity response of neoadjuvant therapy in breast cancer. And E2F1 may be involved in the process of drug resistance by regulating the MAPK signaling pathway. These might be useful as sensitive genes for the efficacy evaluation of neoadjuvant chemotherapy in breast cancer.

## 1. Introduction

Neoadjuvant chemotherapy (NAC) has gained significant attention because of its improved treatment outcome in early breast cancer [1]. NAC therapy can reduce the size of the primary tumor, which eventually increases the rate of breast-conserving therapy and can reduce morbidity [2]. Pathological complete response (pCR) has been established as an intermediate marker for a higher overall survival rate after receiving NAC therapy [3]. Previous studies have shown that some genes show a strong association with pCR and could be considered as important predictors of NAC treatment in breast cancer. For example, hormone receptors [4], the human epidermal growth factor receptor 2 (HER2) [5], and Ki-67 [6] are associated with pCR and could serve as predictors of the response to NAC therapy in breast cancer patients. In addition, it was shown that the high sensitivity to chemotherapy is consistently related to genes that are responsible for various biological pathways of base excision repair (BER), microtubule spindle formation, DNA repair, and cellular aging [7]. Although many studies have investigated the association of genetic factors with pCR, there is still a lot we do not know due to the abundant amount of genes. The microarray or sequencing technology makes it easier for us to investigate the genetic alterations of breast cancer tissues after receiving NAC treatment and to explore its underlying mechanisms.

RETRACTED

A recent sequencing study [8] using digital gene expression profiling analysis compared gene expression profiles of samples from patients presenting pCR with those of samples from patients with nonpathological complete response (NpCR). This sequencing study [8] identified five genes related to the ubiquitin-proteasome pathway (HECTD3, PSMB10, UBD, UBE2C, and UBE2S) and five genes associated with cytokine–cytokine receptor interactions (CCL2, CCR1, CXCL10, CXCL11, and IL2RG), which can be considered as sensitive genes for the efficacy evaluation of the NAC therapy in breast cancer. Parallel to the development of microarray and sequencing technologies, the bioinformatics technique also arose, having many advantages such as the integration and systematic analysis of large amounts of biological information contained in microarray or sequencing studies and the visualization of pathogenic mechanisms through various network analyses. Based on these advantages of bioinformatics analyses on microarray or sequencing studies, it is necessary to use this bioinformatics analysis to include all available microarray or sequencing datasets to comprehensively investigate this topic to the fullest. However, there have so far been no reports on employing a bioinformatic analysis to identify key genes that can predict the sensitivity to NAC therapy in breast cancer.

The aim of this study was focused on the identification of important genetic factors (e.g., genes, transcription factors, and signaling pathways) which can be considered as sensitive predictors of NAC therapy in breast cancer. The genetic mechanisms explored in this study laid the foundation for the development of future chemotherapeutic targeted drugs and also provided direction for future research.

RETRACTED

## 2. Materials and Methods

### 2.1. Cell Lines and Culture

Human breast cancer cells MCF-7 (TCHu 74) were purchased from the National Collection of Authenticated Cell Cultures. The Adriamycin-resistant MCF-7 (MCF-7/ADR) human breast cancer cells were purchased from HAKATA. MCF-7 cells were cultured in High Glucose Dulbecco's Minimum Essential Medium (DMEM, 8120251, Gibco) supplemented with 10% Fetal Bovine Serum (FBS, 40130ES76, YEASEN) and 1% penicillin-streptomycin (15140122, Gibco). The medium used for MCF-7/ADR contained 20% FBS, 1% penicillin-streptomycin, 10 *μ*g/ml insulin (INS, PB180432, Procell), and 20 ng/ml adriamycin (ADR, A1832, APEXBIO). All the cell lines were maintained in a container at 37°C in 5% CO_2_.

### 2.2. Transcriptomic Dataset

The expression profiles related to breast cancer were downloaded from the GEO database, and two publicly available datasets (GSE22226 and GSE21974) were obtained. The GSE22226 dataset was based on two experimental platforms, namely, GPL4133 and GPL1708. This dataset contains 150 samples in total, including 36 samples with pCR after receiving neoadjuvant chemotherapy and 108 samples with non-pCR after receiving neoadjuvant chemotherapy, as well as 6 samples in which the pathological state is unclear. After removing the unclear samples, the GSE22226 dataset was separated into two datasets based on different platforms (GPL4133 and GPL1708). In addition, the GSE21974 dataset was only based on one experimental platform GPL6480 and contained 8 samples with pCR after NAC and 17 samples with non-pCR after NAC treatment. In conclusion, three datasets (GSE22226 under platform GPL4133, GSE22226 under platform GPL1708, and GSE21974 under platform GPL6480) were obtained and included in the analysis.

### 2.3. Differential Expression Analysis

The microarray data of the downloaded expression profiles were background-corrected by using a robust multiarray analysis (RMA) algorithm. After data standardization, the raw probe sequences were converted to genes per the corresponding platform of datasets. The differential expression analysis was performed by using the limma package of the R language. The genes with a *P* value of <0.05 and |log*FC*| ≥ 0.58 were defined as DEGs. The genes with logFC ≥ 0.58 were defined as upregulated genes, while genes with logFC ≤ −0.58 were defined as downregulated genes. The genes which were upregulated in any two datasets were regarded as core upregulated genes, and the genes which were downregulated in any two datasets were regarded as core downregulated genes. After obtaining the DEGs from these three datasets, the numbers of upregulated and downregulated DEGs were counted, respectively.

RETRACTED

### 2.4. Functional Enrichment Analysis

We took the union from the three datasets, meaning that a total of 1917 downregulated genes and 2005 upregulated genes were obtained. The functional enrichment analysis was performed by using clusterProfiler package in R project. The GO_BP analysis was performed to identify the enriched biological processes (BP) by using the enrichGO method in this package; and the KEGG analysis was carried out to identify the enriched signaling pathway by using the enrich KEGG method. The BP and pathways with *P* values of <0.05 were significantly enriched.

### 2.5. Construction of Protein-Protein Interaction Network

The experimentally verified protein-protein interactions (PPIs) were downloaded from the HPRD (Human Protein Reference Database, http://www.hprd.org/). The PPI pairs including core upregulated genes and core downregulated genes were extracted and used to construct a PPI network. The PPI network was constructed and visualized by using the Cytoscape software (version 3.8.0). The topology analysis results can be obtained and exported by clicking Tools-Analyze Network in the GUI option of the software. The topological characteristics of the PPI network were investigated, including degree, betweenness, topological coefficient, and average path length.

### 2.6. Construction of TF-Target Gene Regulatory Network

The transcription factors and their targeted genes were downloaded from three databases including HTRIdb (Human Transcriptional Regulation Interaction, http://www.lbbc.ibb.unesp.br/htri/tf.jsp), TRED (Transcriptional Regulatory Element Database, https://cb.utdallas.edu/cgi-bin/TRED/tred.cgi?process=home), and Genomatix (https://www.genomatix.de/). The TF-gene interaction pairs were integrated, and the TFs among the core upregulated genes and core downregulated genes were extracted and defined as core up-/downregulated TFs. The target genes of these core up-/downregulated TF were obtained. The interaction pairs between core up-/downregulated TFs and their target genes were used for the construction of the core TF-target regulated network. The functional enrichment of core TFs was performed by using the Ingenuity Pathway Analysis (IPA; Ingenuity Systems, http://www.ingenutiy.com).

### 2.7. Predictive Evaluation of Hub TF Genes

The expression values of hub TF genes in three datasets (GSE21974, GSE22226 (GPL1708), and GSE22226 (GPL4133)) were, respectively, obtained to observe the differentially expressed status of these hub TF genes in different datasets. In order to investigate whether the differential expressed results were able to affect the sample types (pCR and non-pCR), the support vector machine (SVM) model was constructed by using scikit-learn package in python. A SVM model was built for each dataset, respectively. 60% of samples in one dataset was regarded as the training set, and 40% of samples in the same dataset was considered to be the test set (Test set 1); meanwhile, the other two datasets were regarded two test sets (Test sets 2 and 3). After building the original model, the GridSearchCV method in scikit-learn was used to identify the best hyperparameter for the model. By setting the CV parameter to be 10 in the GridSearchCV method, the model was able to automatically use 10-fold CV for training. The data was trained by using the SVM model which was optimized by the GridSearchCV method, and the three test sets were predicted. ROC analysis was performed based on the sample scores of the training set and test sets. The performance of the model was evaluated by area under curve (AUC).

RETRACTED

### 2.8. Quantitative Real-Time PCR

The expression of E2F1 and HOXA9 in cells was detected by using quantitative real-time PCR (RT-qPCR). We use Trizol (15596026, Scientific) reagent to extract the total RNAs from the cells. After removing genomic DNA, we use the PrimeScript RT reagent Kit (RR047A, Takara) to reversely transcript RNAs to cDNAs. Then, we added forward and reverse primers of E2F1 and HOXA9 to the samples. Three repeated controls were set in each group. The housekeeping gene glyceraldehyde-3-phosphate dehydrogenase (GAPDH) was used as the internal control. Relative expression of each target gene was normalized to GAPDH mRNA level and calculated with the 2^−*ΔΔ*Ct^ method. The primer sequences used in the PCR are presented in Table 1.

### 2.9. Western Blot

We used RIPA (C874793, MACKLIN) lysate to extract total proteins from MCF-7 and MCF-7/ADR cells and then detect the protein concentration by BCA Protein Assay Kit (20201ES76, YEASEN). The proteins in the lysates were separated by 12% SDS–PAGE Gel (20328ES50, YEASEN); then, we transferred the proteins to PVDF membranes and blocked with 5% skim milk for 1.5 h. After that, we used primary antibodies (9926T, CST) at 4°C to incubate overnight. Finally, we used horseradish peroxidase-conjugated secondary antibody (7076S and 7074S, CST) to incubate 1 h at room temperature. Immunoblots were visualized by the ECL detection system (36208ES60, YEASEN).

## 3. Results

### 3.1. Identification of Up- and Downregulated DEGs

As seen in Table 2, a total of 1182 DEGs were obtained from the GSE21974 dataset, including 661 upregulated DEGs and 521 downregulated DEGs. As for the GSE22226 dataset based on the GPL1708 platform, a total of 238 DEGs were identified, including 132 upregulated DEGs and 106 downregulated DEGs; in the GSE22226 dataset based on GPL4133, a total of 2,605 DEGs were obtained including 1257 upregulated DEGs and 1348 downregulated DEGs. It is observable that one upregulated DEG (KLHDC7B) (shown in Figure 1(a)) and four downregulated DEGs (TFF1, LOC440335, SLC39A6, and MLPH) overlapped in all three datasets (shown in Figure 1(b)).

RETRACTED

### 3.2. Identification of Biological Processes and KEGG Pathways Enriched by DEGs

All the upregulated DEGs obtained from the three datasets were combined, and the same was done for all the downregulated DEGs. The functional enrichment analysis was performed by using the online tools of DAVID (the Database for Annotation, Visualization and Integrated Discovery, https://david.ncifcrf.gov/). This analysis showed that upregulated DEGs mainly regulate some pathways including cell cycle, T cytotoxic cell surface molecules, and steroid biosynthesis (shown in Figure 2(a)); in contrast, the downregulated DEGs mainly regulate some pathways including telomere maintenance, systemic lupus erythematosus, and blood coagulation (shown in Figure 2(b)).

### 3.3. Identification of Core Genes by Constructing a Core Up/Down PPI Network

The DEGs shared by at least two datasets were defined as core genes. 54 core downregulated genes and 44 core upregulated genes were obtained. The experimentally validated PPI pairs of these genes were extracted. The PPI pairs of core down-/upregulated genes were, respectively, used for the construction of a core down PPI network (shown in Figure 3) and a core up PPI network (shown in Figure 4).

After analyzing the topological characteristics of core up/down PPI networks, gene nodes were ranked by their degree in a descending order. In the core down PPI network, the core gene with the highest degree is KRT18, which is followed by MYO5C, WWP1, UQCROQ, PGR, and FOXA1. In the core up PPI network, IL7R has the highest degree, followed by HIST1H1A and E2F1.

### 3.4. Identification of the Four Hub TFs by Constructing a Core TF-Target Regulatory Network

The core transcription factor genes were screened, and their targets were obtained. Three core downregulated TFs (FOXA1, PGR, and SPDEF) and two core upregulated TFs (E2F1 and HOXA9) were screened. By using Cytoscape software, the TF-target regulation network of core up-/downregulated TFs was constructed. The core downregulated TF-target regulation network includes 1081 interaction pairs and 1070 nodes (shown in Figure 5(a)); and the core upregulated TF-target regulation network includes 3580 interaction pairs and 3491 nodes (shown in Figure 6). The highly interconnected module, consisting of three TFs (FOXA1, SPDEF, and PGR) and one gene (CDKN2A) (shown in Figure 5(b)), was extracted from a core downregulated TF-target regulation network, using an MCODE plugin. In this module, three TFs interconnect with each other by directly and indirectly targeting the gene CDKN2A.

RETRACTED

We extracted total RNA from the cells and verified the gene expression levels of E2F1 and HOXA9 by RT-qPCR. We found that E2F1 was low-expressed in MCF-7/ADR compared to MCF-7 but HOXA9 was the opposite (shown in Figures 7(a) and 7(b)).

### 3.5. SVM Models for Evaluating the Classification Performance of Core TFs in Sample Types

Table 3 shows that among the five hub TF genes, 2 genes (i.e., HOXA9 and SPDEF) were differentially expressed in the GSE21974 dataset, 3 genes (i.e., E2F1, FOXA1, and PGR) were differentially expressed in the GSE22226 (GPL1708) dataset, and all of the 5 genes (i.e., E2F1, FOXA1, HOXA9, PGR, and SPDEF) were differentially expressed in the GSE22226 (GPL4133) dataset.

The AUC values of Test One in the GSE21974 dataset and GSE22226 (GPL1708) dataset were, respectively, 61.9% and 70.5% (Figure 8(a) and Figure 8(b)). Such results indicated that there was no significant difference in the expression values of the five TF genes between PCR samples and non-PCR samples; and the SVM model was unable to distinguish the two groups of samples effectively.

In addition, Figure 8(c) shows that the AUC value of Test One in the GSE22226 (GPL4133) dataset was 100%. This result indicated that there is significant difference for the expression values of the 5 TF genes between PCR samples and non-PCR samples; and the SVM model was able to distinguish two groups of samples very well. Such result obtained in the GSE22226 (GPL4133) dataset was exactly consistent with the results regarding the differential expression status of five TFs in the same dataset (Table 4). This finding also indicated that the gene expression values of the five TFs were able to influence the sample types.

We found that the AUC variation of Test Two and Test Three fluctuated greatly (Figures 8(a)–8(c)), and the trained model could not effectively predict the sample types in the other datasets. Based on this reason, another SVM model was built based on the combination of three datasets (Figure 8(d)). Figure 8(d) shows that the SVM based on three datasets had an average prediction performance on test set (AUC = 56.22%), indicating that the pattern of sample expression values in the three datasets was not consistent. Such result might be caused by the differences in terms of sample collecting time, operators, reagent batches, and technical platforms. Based on the above-mentioned results, we concluded that these 5 TF genes have limited influence on the sample types (i.e., pCR and non-pCR). More differential genes might be better for determining the specific sample type.

RETRACTED

### 3.6. The Identification of the Pathways Enriched by Core TFs

For the two core downregulated differentially expressed TFs (FOXA1 and PGR) and two core upregulated differentially expressed TFs (HOXA9 and E2F1), a functional enrichment analysis was performed. The enriched pathways of these core TFs can be seen from Figures 9 and 10. As observed from Figure 9, FOXA1 is mainly involved in pathways including TGF-*β* signaling pathway, signaling by PDGF, and neurotrophin signaling pathway; PGR is mainly involved in pathways including focal adhesion, ECM-receptor interaction, integrin signaling pathway, and MAPK signaling pathway; HOXA9 is mainly involved in pathways including PI3K-Akt signaling pathway, insulin pathway, and chemokine signaling pathway; E2F1 is mainly involved in pathways including cell cycle, p53 signaling, DNA replication, and MAPK signaling.

Next, we detected the expression of several key proteins of the MAPK signaling pathway, such as JNK, p-JNK, p38, Erk, p-Erk, and p-Akt. JNK belongs to protein kinase. After activation, it regulates the proliferation, activation, and metabolism of tumor cells by activating downstream substrates. Wang et al. found that activing the JNK/c-Jun signaling pathway can inhibit colorectal cancer cell proliferation and induce apoptosis [9]. The Erk-MAPK pathway is located downstream of many growth factor receptors, so it is one of the most important for cell proliferation. And Nwosu et al. showed that when metabolism was severely altered in poorly differentiated hepatocellular carcinoma cells, high p-Erk may not indicate higher cell proliferation and that blocking the Erk pathway can lead to increased cell proliferation and resistance [10]. P38 is another important protein in the MAPK signaling pathway. Some studies support that p38, as a tumor suppressor gene [11], can both inhibit cell proliferation and induce apoptosis [12], which plays an antitumor defense role [13]. In addition, many studies showed that overactivation of Akt mediated favor pathways of tumorigenesis and drug resistance [14, 15]. Then, we detected the protein expression of the MAPK signaling pathway mentioned above in two cell lines and found that the pathway was inhibited in MCF-7/ADR (shown in Figure 11). These results suggested that the MAPK signaling pathway might play a role in adriamycin resistance.

RETRACTED

## 4. Discussion

By analyzing and comparing the transcriptional signatures between the pCR group and non-pCR group, many genes, transcription factors, and signaling pathways were identified to be sensitive predictors for chemotherapy response. The underlying mechanisms of these processes in chemotherapeutic drugs targeting breast cancer have been supported by previous scholarly evidence and will be described in this section.

Five DEGs (one upregulated DEG (KLHDC7B) and four downregulated DEGs (TFF1, LOC440335, SLC39A6, and MLPH)) overlapping in three included datasets have been confirmed to be associated with sensitivity for chemotherapy. For example, KLHDC7B (Kelch domain containing 7B, gene ID: 113730) is involved in breast cancer by regulating the interferon signaling pathway, which plays either an immunostimulatory or immunosuppressive role by influencing immune and intrinsic/nonimmune determinants of chemotherapy responses [16, 17]. For another instance, TFF1 (trefoil factor 1; gene ID: 7031) plays a mediating role in the estrogen-promoted resistance to apoptosis induced by doxorubicin in MCF-7 breast cancer cells, indicating that the TFF1 gene could be regarded as a target for augmenting the sensitivity to chemotherapy in breast cancer treatments [18]. In addition, LOC440335 (also called SMIM22 (small integral membrane protein 22); gene ID: 440335) has been examined to be overexpressed in hormone receptor-positive breast tumors. Since the knockout of the gene LOC440335 can lead to a G0/G1 cell cycle arrest [19] and many cytotoxic drugs can inhibit the growth of breast cancer cells by inducing the G0/G1 cell cycle arrest [20], the downregulation of this gene is assumed to be involved in the molecular mechanisms of targeted chemotherapy for breast cancer. Additionally, an investigation studying ductal breast tumor (T47D) cells found that SLC39A6 (solute carrier family 39 member 6; gene ID: 25800) can significantly promote epithelial-to-mesenchymal transition (EMT) [21], which has been defined to be predictive for tumor response following neoadjuvant chemotherapy for breast cancer [22]. Furthermore, MLPH (melanophilin; gene ID: 79083) encodes a member of the exophilic subfamily of Rab effector proteins. The small Rab GTPases acting as essential components of vesicle trafficking machinery have been shown to promote tumor progression [23]. Since targeting vesicle trafficking has been recommended to be a good strategy for cancer chemotherapy [24], dysregulation of the MLPH gene can be assumed to be implicated in the anticancer mechanisms of chemotherapeutic drugs.

RETRACTED

Five transcription factors (HOXA9, SPDEF, FOXA1, E2F1, and PGR) could be regarded as sensitive predictors of chemotherapy response. For example, HOXA9 (homeobox A9; gene ID: 3205) promoter methylation status was related to the response to cisplatin-based neoadjuvant chemotherapy in metastatic bladder cancer [25]. HOXA9 can restrict the progression of breast tumors by regulating the expression of the tumor suppressor gene BRCA1 [26]; however, there have so far been no investigations regarding whether promoter DNA methylation of HOXA9 could be used for predicting response or resistance to neoadjuvant chemotherapy in breast cancer patients. As another example, SPDEF (SAM pointed domain-containing ETS transcription factor; gene ID: 25803) has been demonstrated to be an oncogenic driver and an indicator of poor prognosis in breast cancer [27]. SPDEF can interact with proteins regulating cell cycle, DNA repair, and cytoskeleton organization [28], which can be assumed to be the underlying mechanism of the SPDEF gene being involved in the response to chemotherapeutic agents. In addition, the downregulation of FOXA1 (forkhead box A1; gene ID: 3169) was shown to be associated with a good response to neoadjuvant chemotherapy [29] and could be a prognostic factor related to distant disease-free survival in breast cancer [30]. Additionally, E2F1 (E2F transcription factor 1; gene ID: 1869), as a critical downstream target of the tumor suppressor RB, has been shown to play crucial roles in controlling cell cycle and suppressing proliferation-associated genes [31]. The cell cycle regulating role of E2F1 was also reflected on breast cancer: a previous literature conducted by Hunt et al. showed that the overexpression of E2F-1 promoted apoptosis in human breast carcinoma cell lines [32]. The driving role of E2F1 in chemotherapeutic drug resistance had been well supported by some previous evidence researching various cancers. For example, the upregulation of the E2F1 gene was shown to sensitize osteosarcoma cells to chemotherapeutic drugs [33]. For another example, E2F1 was found to result in chemotherapeutic drug efflux and thus inhibit chemotherapy-induced cell death in lung cancer [34]. Another research regarding colon cancer showed that the ectopic expression of E2F1 allowed the DLD1 colon cancer cell lines to be sensitive to the chemotherapeutic drug cisplatin; however, the knockdown of endogenous E2F1 induced the resistance of colon cancer cell lines to the cytotoxicity of cisplatin [35]. Although E2F1 has been well supported to be involved in chemotherapeutic drug resistance, the functional interplay between the E2F1 gene and chemotherapeutic drugs has not yet been investigated in breast cancer, to the best of the authors' knowledge. Therefore, the current study selected two cell lines (MCF-7 cell lines, as well as adriamycin-resistant MCF-7 cell lines) and verified the expression values of E2F1 in both cell lines. The results of our validation experiments are as expected and shown to be consistent with the expression pattern of E2F1 in previous research [35]: downregulation of E2F1 in drug-resistant cell lines (MCF-7/ADR), while the upregulation of E2F1 in drug-sensitive cell lines (MCF-7). In addition, another identified transcription factor PGR (progesterone receptor; gene ID: 5241) is a hormone receptor gene that can be considered as a classical estrogen receptor (ER) target gene in breast cancer cells [36]. The negativity of PGR expression is a significant predictive factor to achieve pCR after neoadjuvant chemotherapy in HER2-negative breast cancer [37]. Since transcription factors lie at the heart of many fundamental cellular processes (e.g., DNA replication and repair, cell growth and division, and control of apoptosis, as well as cellular differentiation), there is reason to believe that TFs can be responsible for determining the cellular response to chemotherapy; and utilizing cytotoxic drugs to target TFs is, therefore, a promising strategy in the treatment of breast cancer [38].

RETRACTED

In addition, a variety of signaling pathways have been identified to be predictors of chemotherapy response in breast cancer, including pathways related to DNA biosynthesis (e.g., DNA replication, TCA cycle), pathways related to cell cycle (e.g., cell cycle checkpoints, cell cycle mitotic), pathways associated with immune response (e.g., cytokine-cytokine receptor interaction, signaling in the immune system, NO2-dependent IL 12 pathway in NK cells, the role of Tob in T-cell activation, and IL12 and Stat4-dependent signaling pathway in Th1 development), metabolic pathways (e.g., integration of energy metabolism, metabolism of nucleotides, and calcium signaling pathways), and pathways related to angiogenesis (e.g., angiogenesis, signaling by PDGF, blood coagulation, and complement and coagulation cascades). We found that E2F1 was highly expressed in MCF-7, which was consistent with the previous DEG analysis results, so we chose to focus on E2F1. Combined with the analysis results of the E2F1 participation pathway (shown in Figure 9), we decided to study the MAPK signaling pathway, which plays a central role in many cellular signal transduction processes, especially the dual role in cell proliferation and apoptosis [39]. We found that in MCF-7/ADR, the MAPK signaling pathway-related proteins were inhibited, which may promote tumor cell proliferation and inhibited apoptosis, reduce drug efficacy, and led to the production of drug-resistant strains. Therefore, identification of these genes and the MAPK pathway can benefit the treatment of patients, which can be used to increase the efficacy of chemotherapy by synergistically acting with conventional chemotherapeutics.

RETRACTED

Some limitations of this study need to be acknowledged. Firstly, although different subtypes of breast cancer respond distinctly to neoadjuvant therapy with various responses and prognostic values [40], this study did not segregate them into different subtypes. To avoid the complexity of the study design, all subtypes were combined, and investigating the expression alteration of genetic factors between a favorable outcome and adverse outcome was established as the focus of this article. Last but not least, the specific mechanism of the MAPK signaling pathway in the process of cell drug resistance still needs to be further studied. Its proliferation and apoptosis effects in MCF-7/ADR cells need to be verified in many aspects.

In addition, it is important to emphasize the novel discovery as well as the recapitulation of the previous work. Firstly, the current research followed a traditional study design which begins with the prediction of the computational biological analysis and then was followed by the experimental validation to verify the most significant gene or pathway. The innovation of such type of study is that it integrated studies with the same experimental design and thus included bigger sample size, which caused the more accuracy of the results analyzed by integrated multiple studies when compared to the results obtained by individual sequencing or microarray study. Secondly, we found that E2F1 regulates the adriamycin resistance in breast cancer via the MAPK pathway, which has not been reported before. Moreover, many genes (e.g., TFF1, LOC440335, SLC39A6, HOXA9, and FOXA1) identified by the current study have been well evidenced to be related to play driving or regulating roles in tumor chemotherapy drug resistance in the context of breast cancer.

## 5. Conclusion

Neoadjuvant chemotherapy can shrink the tumor and effectively reduce the difficulty and risk of surgery. Therefore, improving the sensitivity of the tumor to neoadjuvant chemotherapy is helpful to improve the therapeutic effect of patients. Our findings suggest that E2F1 is associated with sensitive response and favorable outcome in breast cancer receiving neoadjuvant therapy. We also confirmed that E2F1 was different between common cancer MCF-7 and drug-resistant MCF-7/ADR, and the MAPK signal pathway was inhibited in the MCF-7/ADR cells. These results may guide the development direction of targeted agents which can be incorporated with traditional chemotherapeutic medicine to improve patients' survival.

RETRACTED

## Figures and Tables

**Figure 1:** (a) The shared upregulated DEGs among three datasets. (b) The shared downregulated DEGs among three datasets.

**Figure 2:** (a) The significantly enriched pathways of upregulated DEGs. (b) The significantly enriched pathways of downregulated DEGs.

**Figure 3:** The core down PPI network consisting of interacted genes and core downregulated genes.

**Figure 4:** The core up PPI network consisting of interacted genes and core upregulated genes.

**Figure 5:** The core downregulated TF-target regulatory network: (a) the entire network; (b) the highly interconnected modules in the network.

**Figure 6:** The core upregulated TF-target regulatory network.

**Figure 7:** (a) RT-qPCR analysis of E2F1 mRNA expression in MCF-7 and MCF-7/ADR cells. (b) RT-qPCR analysis of HOXA9 mRNA expression in MCF-7 and MCF-7/ADR cells.

**Figure 8:** The ROC curve analysis results based on SVM models established for different datasets. (a) ROC curves based on the SVM model constructed for the GSE21974 dataset; (b) ROC curves based on the SVM model constructed for the GSE22226 (GPL1708) dataset; (c) ROC curves based on the SVM model constructed for the GSE22226 (GPL4133) dataset; (d) ROC curves based on the SVM model constructed for the combination of three datasets (GSE21974, GSE22226 (GPL1708), and GSE22226 (GPL4133)).

**Figure 9:** The enriched pathways of four TFs: FOXA1 (a), PGR (b), HOXA9 (c), and E2F1 (d).

**Figure 10:** The TF-pathway regulatory network of four TFs (FOXA1, PGR, HOXA9, and E2F1).

**Figure 11:** Western blot analysis suggested the changes of the MAPK signal pathway-related proteins. GAPDH was used as a loading control.

**Table 1:** Primer sequences for PCR.

Gene name	Sequences 5′-3′
E2F1	Forward: CCCATCCCAGGAGGTCACTT
	Reverse: CTGCAGGCTCACTGCTCTC
HOXA9	Forward: GCTTGTGGTTCTCCTCCAGT
	Reverse: CCAGGGTCTGGTGTTTTGTA
GAPDH	Forward: GGAGCGAGATCCCTCCAAAAT
	Reverse: GGCTGTTGTCATACTTCTCATGG

**Table 2:** The number of samples and DEGs obtained from three datasets.

Datasets	Samples			DEGs		
	PCR	nPCR	Total	Up	Down	Total
GSE21974_gene_unique	8	17	25	661	521	1182
GSE22226_GPL1708_unique	32	92	124	132	106	238
GSE22226_GPL4133_unique	4	16	20	1257	1348	2605

**Table 3:** The expression values of 5 hub TF genes in each of the three datasets (GSE21974, GSE22226 (GPL1708), and GSE22226 (GPL4133)), respectively.

Gene	GSE21974		GSE22226 (GPL1708)		GSE22226 (GPL4133)	
	logFC	*P* value	logFC	*P* value	logFC	*P* value
E2F1	-0.474221	0.296375	0.780518	0.000008	0.7886	0.046745
FOXA1	-0.990737	0.218738	-0.929196	0.045423	-2.161614	0.019597
HOXA9	1.52779	0.006588	0.179879	0.397407	1.771187	0.004276
PGR	-0.523549	0.512543	-0.809215	0.002354	-2.63025	0.002446
SPDEF	-1.247146	0.047025	-0.282253	0.140211	-0.854562	0.044214

RETRACTED

**Table 4:** The ROC values of five TFs in each of the three datasets.

Gene	GPL1708	GPL4133	GPL21974
HOXA9	0.5683	0.875	0.8529
SPDEF	0.5863	0.6406	0.7353
FOXA1	0.6325	0.7813	0.6691
E2F1	0.7437	0.8438	0.6176
PGR	0.6637	0.9219	0.5735

## Data Availability

The data that support the findings of this study are available on request from the corresponding author.
